The article "Endothelin-1/Nitric Oxide Ratio as a Predictive Factor of Response to Therapy With Terlipressin and Albumin in Patients With Type-1 Hepatorenal Syndrome" was published in 2020. Journal: Front Pharmacol.

# Endothelin-1/Nitric Oxide Ratio as a Predictive Factor of Response to Therapy With Terlipressin and Albumin in Patients With Type-1 Hepatorenal Syndrome

**DOI:** 10.3389/fphar.2020.00009

**Published:** 2020-01-31

**Authors:** Ahmed Abdel-Razik, Nasser Mousa, Mostafa Abdelsalam, Ahmed Abdelwahab, Mona Tawfik, Ahmed M. Tawfik, Ahmad S. Hasan, Rania Elhelaly, Niveen El-Wakeel, Waleed Eldars

**Affiliations:** ^1^ Tropical Medicine Department, Faculty of Medicine, Mansoura University, Mansoura, Egypt; ^2^ Nephrology and Dialysis Unit, Internal Medicine Department, Faculty of Medicine, Mansoura University, Mansoura, Egypt; ^3^ Diagnostic & Interventional Radiology Department, Faculty of Medicine, Mansoura University, Mansoura, Egypt; ^4^ Clinical Pathology Department, Faculty of Medicine, Mansoura University, Mansoura, Egypt; ^5^ Medical Microbiology and Immunology Department, Faculty of Medicine, Mansoura University, Mansoura, Egypt

**Keywords:** hepatorenal syndrome, endothelin-1, nitric oxide, liver cirrhosis, endothelin-1/nitric oxide ratio, terlipressin, albumin

## Abstract

**Background and Purpose:**

Predictors of response to type-1 hepatorenal syndrome (HRS) therapy are urgently needed. This study's purpose is to evaluate the proposed predictors in these patients.

**Methods:**

Forty-two type-1 HRS patients with cirrhosis were treated with albumin and terlipressin. Clinical, biochemical, and demographic parameters taken at the onset of therapy and changes in endothelin-1/nitric oxide (ET-1/NO) ratio during therapy were analyzed to check their predictive value.

**Results:**

Response to treatment (serum creatinine level <1.5 mg/dL at the end of therapy) was shown in 20 patients (48%). Independent predictive variables of response to therapy were early reduction of ET-1/NO ratio ≥0.15 at day 3 of therapy and serum bilirubin baseline <8 mg/dL (area under the receiver operating characteristic curve, 0.751; *P* < 0.001; specificity, 55%; sensitivity, 85%). Response rates in patients with serum bilirubin level <8 and ≥8 mg/dL were 63% and 20%, respectively (*P* = 0.008). The corresponding values in patients with an early reduction of ET-1/NO ratio ≥0.15 and <0.15 on day 3 were 85% and 13.6%, respectively (*P* < 0.001).

**Conclusions:**

Early reduction of ET-1/NO ratio and lower serum bilirubin baseline can predict response to type-1 HRS therapy with albumin and terlipressin. Alternative therapy should be investigated for nonresponder type-1 HRS patients.

## Introduction

Hepatorenal syndrome (HRS) is a reversible cause of renal impairment that occurs in patients with cirrhotic ascites, as well as in patients with alcoholic hepatitis or acute liver failure who show no significant abnormalities in the kidneys morphology (Arroyo et al., 1996; Dagher and Moore, 2001; Angeli et al., 2015).

The article "Endothelin-1/Nitric Oxide Ratio as a Predictive Factor of Response to Therapy With Terlipressin and Albumin in Patients With Type-1 Hepatorenal Syndrome" was published in 2020. Journal: Front Pharmacol.

HRS is characterized by marked alterations in cardiovascular function, impaired renal function, and over-activity of renin-angiotensin systems that lead to severe renal vasoconstriction with a significant reduction of the glomerular filtration rate (GFR) as well as vigorous activation of the sympathetic nervous system (Arroyo et al., 1996; Dagher and Moore, 2001).

HRS predicts mortality in cirrhosis. The most important aspect of providing care to patients with HRS is an evaluation of candidacy for orthotopic liver transplantation (Gonwa et al., 1995; Jeyarajah et al., 1997; Nair et al., 2002). Current accessible therapies other than liver transplantation for HRS consist of albumin and the utilization of vasoconstrictors, for example, terlipressin (Angeli and Merkel, 2008).

Recently, only 52% of HRS patients have responded to therapy with terlipressin (Møller et al., 2000; Fabrizi et al., 2006; Gluud et al., 2010; Allegretti et al., 2017). Furthermore, few researches have reported some predictors of response to treatment in HRS patients treated with this regimen.

The endothelium release many vasoactive mediators that change the structure and function of the vascular smooth muscle in response to mechanical and humoral stimuli. Two of the most prominent are ET and NO (Cahill et al., 2001). ET-1 is released in response to infectious complications with an inflammatory response in the form of transcription mediators activation and proinflammatory cytokines (IL-1, IL-6, and TNF-α) production. It also plays an important role in the vascular disruption pathogenesis caused by infection (Charpin et al., 2001; Yeager et al., 2012; Freeman et al., 2014).

The pathophysiology of various disorders is closely related on the ET-1/NO imbalance (Alonso and Radomski, 2003). In cirrhosis and HRS, the ET system dysfunction causes hemodynamic disturbances (Moore et al., 1992; Uchihara et al., 1992).

The identification of patients with low therapeutic response probability is of imperative clinical importance, especially in patients waiting for transplantation. In our study, we evaluated the hypothesized predictors of response to albumin and terlipressin in type-1 HRS and cirrhosis patients treated with this protocol.

## Patients and Methods

### Study Population

Starting 2015, patients with renal impairment and cirrhosis admitted to the Tropical Medicine Department (Mansoura, Egypt) were assessed using the same diagnostic algorithm (Gine`s et al., 2003), that involves evaluation of the possible causes of hypovolemia, diuretic withdrawal, possible infection, drug nephrotoxicity, and renal parenchymal disorders. To exclude the presence of volume depletion related renal failure, plasma expansion with I.V. albumin was tried. According to the International Ascites Club (Arroyo et al., 1996), patients who met the type-1 HRS criteria, were treated with albumin and terlipressin. The new HRS defining criteria were approved by this study protocol (Angeli et al., 2015). Some patients didn't receive therapy due to having advanced hepatocellular carcinoma, severe cardiovascular disorders and/or being terminal cases (death expected in less than 2 days).

The article "Endothelin-1/Nitric Oxide Ratio as a Predictive Factor of Response to Therapy With Terlipressin and Albumin in Patients With Type-1 Hepatorenal Syndrome" was published in 2020. Journal: Front Pharmacol.

All the differential diagnosis causes of cirrhotic acute kidney injury including: organic (including glomerulonephritis and acute tubular necrosis), prerenal (all accessible hypovolemic causes), and obstructive nephropathy (Garcia-Tsao et al., 2008; Møller et al., 2014) were excluded in this study by meticulous history taking and physical examination, together with complete biochemical analysis and radiological investigations.

The existence of infection was assessed by various methods, for example, culture and sensitivity testing for ascitic fluid, blood, sputum, and urine, evaluation of the ascitic fluid absolute polymorphonuclear (PMN) count, and chest radiography. Patients with infection were precluded from this study and received albumin and terlipressin only when renal failure continued after the infection was successfully treated. According to the type of infection, bacterial infections were initially treated with antibiotics as reported in detail elsewhere (Martin-Llahi et al., 2011; Fernandez et al., 2012). The antibiotic was changed according to the results of the cultures if there was no response to the initial therapy. In patients with negative cultures and not responding to the initial therapy, empiric antibiotics policy consisting of vancomycin and carbapenems combination was used (Barreto et al., 2014).

The current study included 42 consecutive cirrhosis/type-1 HRS patients who were subjected to treatment from March 2015 to February 2019. Twenty nine (69%) of them had bacterial infection induced type-1 HRS including 20 SBP cases, six soft tissue infection cases, and three patients with pneumonia as well as 13 patients with HRS without known risk factors.

Bacterial infections were categorized according to the following criteria: SBP is the presence of an ascitic ﬂuid absolute polymorphonuclear count >250/mm^3^ and/or a positive ascitic fluid bacterial culture with no apparent source of infection (Rimola et al., 2000); spontaneous bacteremia is positive blood cultures without an evident source of infection; local infections (skin infection, urinary tract infection, pneumonia, gastroenteritis, meningitis, and biliary tract infection) were evaluated utilizing standard criteria; sepsis with negative-culture is leukocytosis with/without band forms, the presence of fever (>38°C), together with negative cultures, after the exclusion of disorders other than infection that could be related to the systemic inﬂammatory response.

The article "Endothelin-1/Nitric Oxide Ratio as a Predictive Factor of Response to Therapy With Terlipressin and Albumin in Patients With Type-1 Hepatorenal Syndrome" was published in 2020. Journal: Front Pharmacol.

Improvement of SBP was deﬁned as a reduction in polymorphonuclear cell count <250/mm^3^, absence of clinical signs of infection, negative cultures, and normal leukocyte count. The remaining infections were improved according to the conventional criteria. Septic shock was identified as a mean arterial pressure below 60 mmHg regardless of adequate volume resuscitation and need for vasopressor agents (Dellinger, 2003).

In this study, all specific therapy or treatment was delayed for type-1 HRS until the infection has been cured.

In addition, the control group included 42 cirrhotic patients without renal impairment who were sex- and age-matched subjects (male/female = 27/15).

### Treatment Protocol

The response to treatment was considered a primary endpoint, determined by either a decline in serum creatinine level >50% of the pretreatment value, or >1.5 mg/dL during treatment with an end-of-therapy level of ≤1.5 mg/dL.

Terlipressin (Glypressin, Ferring S.A., Saint-Prex, Switzerland) was administrated as follows; 0.5–1 mg/4 h, as intravenous (i.v.) bolus for 3 days with an increase up to 2 mg/4 h for those whose values did not decrease by at least 25% of the pretreatment values. The maximum duration of therapy was 2 weeks. Once serum creatinine is reduced below 1.5 mg/dL, Terlipressin was withheld. If patients developed manifestations matching the ischemic complications, administration of Terlipressin was stopped.

All patients received albumin (Baxter Human Albumin 20%, Baxter AG, Industriestraße 67, A-1221 Vienna, Austria) at a dose of 1 g/kg BW. during the first day, followed by 40 g/d, given for a maximum of 15 days, in order to reach the inferior vena cava collapsibility index (*IVCCI*) ≥40% and ≤75%. Clinically, *IVCCI* was evaluated daily in a regular manner throughout the follow-up period. The dose of albumin was decreased to 20 g/d and/or was stopped if *IVCCI* was <40% (Brennan et al., 2006). All measurements were carried out by qualified ultrasound radiologists. Moreover, if radiological and clinical signs of pulmonary edema developed, the administration of albumin was withheld, and the patients received i.v. doses of furosemide with careful follow-up.

During therapy of HRS, any complications of cirrhosis were treated based on standardized therapeutic measures (Cardenas and Gine`s, 2005).

The article "Endothelin-1/Nitric Oxide Ratio as a Predictive Factor of Response to Therapy With Terlipressin and Albumin in Patients With Type-1 Hepatorenal Syndrome" was published in 2020. Journal: Front Pharmacol.

### Sampling

Following an overnight fasting of 12 h, 4 to 8 mL blood *were withdrawn* through cannulas in superficial forearm *veins* for all patients [1 mL in EDTA for complete blood count (CBC), 5mL without anticoagulants for serum samples].

### Methodology

CBC was assessed using the CELL-DYN Emerald cell counter (Abbott, Wiesbaden, Germany). Serum creatinine, blood urea nitrogen (BUN) and liver function tests were measured on a Dimension Xpand plus chemistry analyzer (Siemens Technology, Princeton, NJ, USA) using commercially available enzyme-based kit and reagents. Quantitative detection of plasma nitric oxide (NO) was measured using ELISA kits provided by MyBiosource (San Diego, CA 92195-3308, USA) Cat No. MBS264607, with detection range 1.56 to 100 nmol/mL (nmol/mL = µmol/L). Though the NO role in various disorders is debatable, the majority of researchers agree that evaluating serum levels of NOx are associated with NO production. (Andrukhov et al., 2013). Quantitative detection of plasma Endothelin-1 (ET-1) was measured using ELISA kits provided by MyBiosource (San Diego, CA 92195-3308, USA) Cat No. MBS025621, with detection range 6.25 to 200 pg/mL (pg/mL = ng/L). Plasma L-Arginine was quantitatively measured using ELISA kits provided by ALPCO (26G Keewaydin Drive, Salem, New Hampshire 3079, United States) Cat No. 30-7733, with detection range 12.5 to 300 µmol/L. The estimated glomerular filtration rate (eGFR) was calculated according to the following formula (Levey et al., 1999): 186 x (Creatinine/88.4)^-1.154^ x (Age)^-0.203^ x (0.742 if female) x (1.210 if black). The ET-1/NO ratio was calculated and recorded for all patients.

### Ethics

The protocol of this study was completed to acclimate with the Declaration of Helsinki and was affirmed by the Ethics Committee of the Mansoura University. Informed consent was obtained from all enrolled patients or their legal representatives.

### Statistical Analysis

The analysis was carried out using SPSS version 20 for Windows (SPSS Inc., Chicago, IL). Results are expressed as the mean ± SD. Comparisons of continuous and categorical variables between patients were carried out using Student *t*- and *X* ^2^-tests respectively. A paired Wilcoxon test and Student *t*-test were used to compare the variables measured at various time points. The multivariate analysis was built using the univariate analysis parameters that had a significant predictive value (*P* < 0.01). The best cutoff values for variables with independent predictive value were measured using receiver operating characteristic curves. The probability of response was evaluated using the Kaplan–Meier method. The calculation of overall response involved patients who received a liver transplant (n = 3) and the results were viewed redacted at the time of transplantation. *P* < 0.05 was considered statistically significant.

The article "Endothelin-1/Nitric Oxide Ratio as a Predictive Factor of Response to Therapy With Terlipressin and Albumin in Patients With Type-1 Hepatorenal Syndrome" was published in 2020. Journal: Front Pharmacol.

## Results

### Patient Characteristics

Only 42 out of the 121 patients with cirrhotic ascites and renal failure were included in this study. The etiology of renal failure was evaluated after admission and HRS was diagnosed following the diagnostic criteria reported by Angeli et al. Of all the excluded patients, 51 were due to previous infection exposure who were discharged from hospital with normal renal function after adequate therapy of infection (32 SBP, 12 soft tissue infections and 7 pneumonia), six due to nephrotoxic agents administration (four aminoglycosides and two contrast agents), seven due to hypovolemic causes (five GIT bleeding and two severe vomiting), and three due to obstructive nephropathy. Also, the 12 patients who showed complete response and marked serum creatinine decline after receiving only albumin as a corrective measure for the pre-renal causes of renal failure were excluded.

Baseline characteristics of patients with type-1 HRS at the time of diagnosis before starting the treatment with albumin and terlipressin are reported in **Table 1**. Not surprisingly, most patients with type-1 HRS had severe liver failure, as demonstrated by increased international normalized ratio (INR), high Model for End-Stage Liver Disease (MELD) and Child-Pugh scores, low estimated GFR using Modification of Diet in Renal Disease equation, high levels of serum bilirubin, creatinine, L-arginine, NOx, serum ET-1, and ET-1/NO ratio *compared* to the control group.

**Table 1:** Baseline characteristics of patients with type-1 hepatorenal syndrome at the time of diagnosis.

Parameters	Cirrhotic patients with HRS (n = 42)	Cirrhotic patients without HRS (control group) (n = 42)	*P*
Age (years)	45 ± 9	44 ± 8.7	0.61
Sex (male/female)	29/13	27/15	0.889
BMI (kg/m^2^)	27 ± 5.9	26.5 ± 5.4	0.686
Etiology of liver cirrhosis			
CHB-related liver cirrhosis	39 (92.8)	37 (88.1)	0.466
CHB-related liver cirrhosis	2 (4.8)	3 (7.2)	0.645
NASH-related liver cirrhosis	1 (2.4)	2 (4.7)	0.571
Hematocrit (%)	28 ± 7	30 ± 8.5	0.243
WBCs (×10^3^/mm^3^)	4.7 ± 2.4	4.5 ± 2.1	0.686
Platelet count (×10^3^/mm^3^)	95 ± 74	102 ± 69	0.655
AST (U/L)	60 ± 32	56 ± 27	0.538
ALT (U/L)	55 ± 27	50 ± 24	0.372
T. Bilirubin (mg/dL)	10.8 ± 8.3	1.9 ± 1.2	<0.001
Serum albumin (g/dL)	2.6 ± 0.6	2.5 ± 0.7	0.484
INR	2.2 ± 0.6	1.8 ± 0.5	0.001
Serum creatinine (mg/dL)	2.8 ± 1.4	1.1 ± 0.4	<0.001
eGFR (mL/min/1.73 m^2^)	57 ± 2.9	74 ± 9.3	<0.001
BUN (mg/dL)	38.4 ± 8.4	37.7 ± 7.9	0.695
Urine volume (mL/d)	585 ± 279	968 ± 453	<0.001
Na (mmol/L)	129 ± 7	130 ± 11	0.621
K (mmol/L)	4.12 ± 0.7	4.23 ± 0.8	0.504
Child-Pugh score	11+1.5	9.75+1.3	<0.001
MELD score	28 ± 9	22+10	0.005
L-arginine (μmol/L)	92.5 ± 15.3	74.5 ± 10.2	<0.001
Oxide metabolites (NOx) (μmol/L)	70.6 ± 3.9	49.5 ± 1.1	<0.001
Endothelin-1 (ET-1) (ng/L)	29.1 ± 1.9	13.3 ± 0.9	<0.001
ET-1/NO ratio	0.42 ± 0.036	0.27 ± 0.02	<0.001

BMI, basal metabolic index; CHB, chronic hepatitis B; CHC, chronic hepatitis C; eGFR, estimated glomerular filtration rate; MELD score, Model for End-Stage Liver Disease score; NASH, nonalcoholic steatohepatitis; WBCs, white blood cells; ALT, alanine aminotransferase; AST, aspartate aminotransferase; INR, international normalized ratio; Na, sodium; K, potassium; ET-1/NO ratio, endothelin-1/nitric oxide ratio.

The article "Endothelin-1/Nitric Oxide Ratio as a Predictive Factor of Response to Therapy With Terlipressin and Albumin in Patients With Type-1 Hepatorenal Syndrome" was published in 2020. Journal: Front Pharmacol.

### Predictive Factors For Treatment Response

Twenty out of the 42 patients (48%) had a response to therapy. Generally, at the end of therapy, serum creatinine decreased below 1.5 mg/dL, while in two patients serum creatinine decreased >50% of the pretreatment levels but stayed above 1.5 mg/dL (4.8 decreased to 1.8 mg/dL and 3.7 to 1.7 mg/dL). The rest of the patients (52%) failed to reach the response to therapy criteria. Serum creatinine levels during the therapy period in non-responders and responders are summarized in **Figure 1**. During therapy, the probability of response in all patients is shown in **Figure 2**. The estimated period for response was approximately 2 weeks. Response to therapy was merely constant in most patients. Recurrence of HRS was 4/20 (20%) in patients who responded to therapy. The average period for recurrence was 2 weeks (range, 3–38 days).

**Figure 1:** Changes in serum creatinine concentration during treatment in responders and nonresponders.

**Figure 2:** Probability of response to treatment in patients with type 1 HRS treated with albumin and terlipressin. Dotted lines represent 95% confidence intervals. The numbers under the curve are patients at risk at each time.

At baseline, several parameters obtained were assessed for the predictive value of response to therapy (**Table 2**). Parameters related to response to therapy (*P* < 0.05) were WBCs count, AST level, serum bilirubin level, urine volume, and MELD score. Furthermore, neither ET-1/NO ratio nor serum creatinine level at baseline was related to response to treatment. The only parameter found to have an independent predictive value in the multivariate analysis was the serum bilirubin level (OR, 14.2; 95% CI, 1.256–160.77; *P* = 0.032). By receiver operating characteristic curves, serum bilirubin level has a cutoff value (< 8 mg/dL) that well-predicted response to therapy, (AUC = 0.751; *P* < 0.001; specificity = 55%; sensitivity = 85%; PPV = 63%; and NPV = 80%). Response rates in patients classified based on baseline serum bilirubin level <8 or ≥8 mg/dL were 63% (17/27) and 20% (3/15), respectively (*P* = 0.008).

The article "Endothelin-1/Nitric Oxide Ratio as a Predictive Factor of Response to Therapy With Terlipressin and Albumin in Patients With Type-1 Hepatorenal Syndrome" was published in 2020. Journal: Front Pharmacol.

**Table 2:** Univariate analysis of baseline parameters according to response to treatment with albumin and terlipressin.

Parameters	Responders (n = 20)	Non-responders (n = 22)	*P*
Age (y)	44 ± 10	43 ± 8	0.72
Sex (male/female)	14/6	15/7	0.97
BMI (kg/m^2^)	25 ± 5.2	27 ± 6.1	0.26
Etiology of liver cirrhosis			
CHC-related liver cirrhosis	19 (95)	20 (91)	0.62
CHB-related liver cirrhosis	1 (5)	1 (4.5)	0.94
NASH-related liver cirrhosis	-	1 (4.5)	-
Hematocrit (%)	27 ± 6	29 ± 8	0.37
WBCs (×10^3^/mm^3^)	4.1 ± 2.2	5.8 ± 2.7	0.03
Platelet count (×10^3^/mm^3^)	108 ± 85	91 ± 69	0.48
AST (U/L)	49 ± 27	69 ± 34	0.04
ALT (U/L)	48 ± 23	63 ± 31	0.08
T. bilirubin (mg/dL)	5.5 ± 1.8	15.5 ± 9	<0.001
Serum albumin (g/dL)	2.5 ± 0.7	2.6 ± 0.8	0.67
INR	1.9 ± 0.6	1.8 ± 0.5	0.56
Serum creatinine (mg/dL)	2.3 ± 1.4	2.9 ± 1.6	0.21
eGFR (mL/min/1.73 m^2^)	58 ± 2.5	56 ± 2.7	0.02
BUN (mg/dL)	38 ± 8.2	38.7 ± 8.8	0.792
Urine volume (mL/d)	475 ± 125	395 ± 90	0.02
Na (mmol/L)	129 ± 9	126 ± 7	0.23
K (mmol/L)	4 ± 0.9	4.11 ± 1	0.71
Child-Pugh score	11 ± 1	12 ± 2	0.051
MELD score	20 ± 6	25 ± 9	0.04
L-arginine (μmol/L)	89.4 ± 12.4	84.5 ± 11.3	0.19
Oxide metabolites (NOx) (μmol/L)	72 ± 2.8	69.5 ± 4.9	0.052
Endothelin-1 (ET-1) (ng/L)	29.7 ± 1.2	30.5 ± 1.4	0.055
ET-1/NO ratio	0.43 ± 0.016	0.44 ± 0.028	0.169

BMI, basal metabolic index; CHB, chronic hepatitis B; CHC, chronic hepatitis C; eGFR, estimated glomerular filtration rate; MELD score, Model for End-Stage Liver Disease score; NASH, nonalcoholic steatohepatitis; WBCs, white blood cells; ALT, alanine aminotransferase; AST, aspartate aminotransferase; INR, international normalized ratio; Na, sodium; K, potassium; ET-1/NO ratio, endothelin-1/nitric oxide ratio.

Based on changes in the ET-1/NO ratio evaluated at day 3 of therapy, we analyzed response rates in all patients. The value of the ET-1/NO ratio used was the average value of all measurements of ET-1/NO ratio assessed at day 3; a reduction in ET-1/NO ratio of 0.15 was considered relevant and used as a cutoff value. Values of ET-1/NO ratio throughout therapy in non-responders and responders are summarized in **Figure 3**. Although the baseline ET-1/NO ratio was not a predictive factor of response, early changes of ET-1/NO ratio within the first days of therapy predicted response. Patients with a reduction in the ET-1/NO ratio equal to or greater than 0.15 at day 3 of therapy had a response rate at the end of treatment of 85% (17/20) compared to 13.6% (3/22) in patients with minimal decreases in the ET-1/NO ratio (*P* < 0.001). When this decrease in the ET-1/NO ratio of 0.15 or more at day 3 was enclosed in the multivariate analysis with the baseline parameters, the predictive factors of response to treatment were the baseline serum bilirubin level and the decrease in the ET-1/NO ratio ≥0.15 at day 3 (**Table 3**). Moreover, 2/5 patients (40%) responded if there was a reduction ET-1/NO ratio ≥0.15 in those with baseline serum bilirubin level ≥8 mg/dL, compared to a response in 1/10 (10%) in those with a change in the ET-1/NO ratio <0.15 with baseline serum bilirubin level ≥8 mg/dL (**Figure 4**).

The article "Endothelin-1/Nitric Oxide Ratio as a Predictive Factor of Response to Therapy With Terlipressin and Albumin in Patients With Type-1 Hepatorenal Syndrome" was published in 2020. Journal: Front Pharmacol.

**Figure 3:** Changes in ET-1/NO ratio during treatment in responders and nonresponders.

**Table 3:** Parameters with independent predictive value of response to treatment with albumin and terlipressin in patients with type 1 HRS.

Parameters	Univariate analysis			Multivariate analysis		
	OR	95% CI	*P*	OR	95% CI	*P*
Baseline serum bilirubin	6.8	1.54–30.8	0.012	14.2	1.256–160.77	0.032
∆ ET-1/NO ratio at day 3 ≥1.5	35.9	6.37–202.2	< 0.001	59.3	5.98–586.92	< 0.001
∆ Serum creatinine at day 3 > 0.5 mg/dL	5.0	1.35–18.6	< 0.001	9.46	0.84–105.9	0.048

CI, confidence interval; OR, odds ratio; ET-1/NO ratio, endothelin-1/nitric oxide ratio.

**Figure 4:** Response rate according to levels of ET-1/NO ratio and its relationship to serum bilirubin at baseline.

In addition, Spearman's correlation analysis showed that there was a significant correlation between the ET-1/NO ratio and serum bilirubin level, serum creatinine level, creatinine clearance, MELD and Child-Pugh scores (*rho* = 0.63, *P* < 0.001; *rho* = 0.72, *P* < 0.001; *rho* = −0.66, *P* < 0.001; *rho* = 0.72, *P* < 0.001; *rho* = 0.69, *P* < 0.001respectively).

During therapy, the early decrease in serum creatinine was also used as a predictor of response to treatment. Response to therapy was demonstrated in 15 of the 19 patients (79%) in whom serum creatinine decreased by at least 0.5 mg/dL at day 3, compared to only 5 of the 23 patients (22%) in whom serum creatinine did not decrease 0.5 mg/dL or elevated at day 3 compared to the baseline (*P* < 0.001). When the cutoff value for the change in serum creatinine used was 1 mg/dL instead of 0.5 mg/dL similar figures were demonstrated (89% and 36%, respectively; *P* = 0.005). The value of the reduction in serum creatinine at day 3 as a predictor of response to treatment was also approved in the multivariate analysis model (odds ratio, 9.46; *P* = 0.048).

### Complications of Cirrhosis

A total of 47 major cirrhotic complications were developed in 37 patients (88%) during therapy: 32 patients with hepatic encephalopathy, five patients with GIT bleeding, and ten patients with bacterial infection. Bacterial infections between responders and non-responders showed no signiﬁcant difference [4/20 (20%) vs. 6/22 (27%), respectively; *P* = 0.6]. The median value for WBCs count was 7,100/mm^3^ and throughout therapy, the occurrence of bacterial infections was partially more common in patients higher count than in those with lower count [7/23 (30.4%) vs. 3/19 (15.8%), respectively; *P* = 0.275]. At the lower WBCs count baseline, patients acquired pneumonia (n = 1) and urinary tract infections (n = 2) after an average period of 6 days (range, 2–10 days), while at the higher WBCs count baseline, patients acquired pneumonia (n = 2) and sepsis (n = 5) after an average period of 6 days (range, 2–14 days).

The article "Endothelin-1/Nitric Oxide Ratio as a Predictive Factor of Response to Therapy With Terlipressin and Albumin in Patients With Type-1 Hepatorenal Syndrome" was published in 2020. Journal: Front Pharmacol.

### Side Effects of Therapy

Eight patients (19%) developed albumin/terlipressin therapy-related side effects. Signs of circulatory overload developed in four patients, that improved after short-lived cessation of albumin but not of terlipressin and furosemide was added in small doses. Intestinal ischemia signs developed in two patients, that disappeared after cessation of therapy. Transient arrhythmia (ventricular extrasystolia) developed in two patients, that did not need persistent cessation of therapy, and improved after therapy withdrawal. We followed up with the patients for at least 3 months after their hospital discharge.

### Survival

90 days after the initiation of treatment, 32 (76.2%) patients died, 6 (14.3%) patients were still alive, 3 (7.2%) participants had undergone liver transplantation, and 1 (2.4%) patient was lost to follow-up as well as the survival probability at that time was significantly higher in responders (40%) with median survival of 65 days compared to non-responders (9%) with median survival of 8 days; *P* < 0.001). Septic shock (n = 16), multiorgan failure (n = 11), liver failure (n = 4), and/or unknown (n = 1) were the *causes of death.*

Using the original MELD risk equation, Area Under the Receiver Operating Characteristic Curve (AUROC) analysis revealed that a MELD score threshold of 20 corresponded to median survival less than 3-months (**Figure 5**). Kaplan-Meier survival curves of patients stratified by baseline MELD score below or above 20, which represents threshold for 3-month median survival. Median survival of patients with baseline MELD score <20 significantly greater than those with baseline MELD scores ≥ 20 (62 vs. 15 days, *P* < 0.001).

**Figure 5:** Kaplan-Meier survival curves of patients stratified by baseline MELD score below or above 20, which represents threshold for 3-month median survival. Median survival of patients with baseline MELD score <20 significantly greater than those with baseline MELD scores ≥ 20 (62 vs. 15 days, *P* < 0.001).

The article "Endothelin-1/Nitric Oxide Ratio as a Predictive Factor of Response to Therapy With Terlipressin and Albumin in Patients With Type-1 Hepatorenal Syndrome" was published in 2020. Journal: Front Pharmacol.

## Discussion

This recent study reports that albumin with terlipressin are currently the accepted therapy for type-1 HRS, but over 50% of patients show a suboptimal to no response to treatment (Dagher and Moore, 2001; Angeli et al., 2015). It is therefore of paramount importance that we keep searching and investigating not only for adequate predictors of response but also prognostic factors before beginning the treatment or early afterward. Obviously, patients responding to treatment showed a statistically significant decline in ET-1/NO ratio at the end of therapy; probably because the low effective arterial blood volume of HRS was improved. These outcomes firmly recommend that the gainful impact of terlipressin in the treatment of HRS is identified with its ability to enhance systemic hemodynamics (Fabrizi et al., 2006; Moreau and Lebrec, 2006). We still don't know why in some type-1 HRS patients the systemic hemodynamics were not enhanced when treated with terlipressin. This may be due to the presence of concomitant adrenal insufficiency, and latent infections associated with higher levels of ET-1 (Hocher et al., 1999).

Independent predictors of response to treatment were serum bilirubin levels at baseline and a decline in the ET-1/NO ratio ≥0.15 at day 3 of therapy. Eleven of the eleven patients (100%) with serum bilirubin at baseline <8 mg/dL who demonstrated a decline in the ET-1/NO ratio ≥0.15 at day 3 responded to our therapeutic protocol. While only one of the 10 (10%) patients with serum bilirubin at baseline ≥8 mg/dL and a reduction in the ET-1/NO ratio <0.15 had a response to therapy. In previous studies, predictive variables of response observed in patients with HRS involved MELD and Child-Pugh scores, arterial pressure, and serum creatinine level at the baseline (Moreau et al., 2002; Alessandria et al., 2007; Neri et al., 2008; Sanyal et al., 2008; Sharma et al., 2008). But some drawbacks may be observed as a small number of patients received therapy as well as analysis may have involved patients treated with different vasoconstrictors e.g. norepinephrine instead of terlipressin.

The association between the renal response to terlipressin and the presence of an early reduction of the ET-1/NO ratio shows the significance of the enhancement of systemic hemodynamics in accomplishing type-1 HRS reversal. ET-1 and NO are the most important local vasoconstrictor and vasodilator respectively. They seem to play a role in almost every tissue and organ (Hei et al., 2006). Recent researches reported that the important factors in identifying the harmful versus beneficial effects of NO are the site of NO production, duration of action, and its amount (Hon et al., 2002). It has been proposed that the disequilibrium of ET-1 and NO levels may have an impact on the pathophysiology of local and systemic circulation disorders. This imbalance in the renal microcirculation has been proposed to be in charge of the dynamic disintegration in kidney function in these patients and the development of HRS (Kayali et al., 2009).

The article "Endothelin-1/Nitric Oxide Ratio as a Predictive Factor of Response to Therapy With Terlipressin and Albumin in Patients With Type-1 Hepatorenal Syndrome" was published in 2020. Journal: Front Pharmacol.

ET-1 may be involved in both impaired glomerular perfusion and renal vasoconstriction which causes HRS (Moore, 2004). Renal blood flow is not the only factor contributing to changes in glomerular filtration rate as seen at the microcirculatory level. The enhanced production of vasoactive mediators including ET-1 causes reduction of the surface area available for glomerular filtration and contraction of mesangial cells which contributes to this phenomenon (Ring-Larsen, 1977; Simonson and Dunn, 1990). The intake of ETA and ETB receptors antagonists combination prevented and in sometimes reversed the pathogenesis of renal failure in different experiments (Anand et al., 2002). Physiologically, early reduction of the ET-1/NO ratio is considered a good prognostic marker in HRS patients with end stage liver disease or on the liver transplantation waiting list.

Interestingly, serum bilirubin level at baseline was considered an independent predictive factor of response to treatment. Poor response to therapy and elevated serum bilirubin levels association can't be explained, but looks to be unrelated to the hemodynamic response to terlipressin. The mechanisms explaining the lack of response to terlipressin related to high serum bilirubin levels are interesting and merits examination. The correlation between the ET-1/NO ratio and bilirubin noticed in this study demonstrates that the values of ET-1 are influenced by the excretory liver function. A correlation between ET-1 and bilirubin has been approved also by some (Nozue et al., 1995; Bachmann-Brandt et al., 2000), but not all authors (Isobe et al., 1993). The possible explanation, not determined by our data, maybe owing to indirect (excess pulmonary *arteriovenous* shunts that increased with the deterioration of liver condition) and direct (reduced clearance of ET-1 by the hepatic tissue) associations. Leakage of bile into the blood and/or disturbance of ET-1 degradation may result in increased serum ET-1 levels since ET-1 is excreted through the biliary system (Cai et al., 1999).

The multivariate analysis model showed that the reduction in serum creatinine level at day 3 can be considered a predictor of response to treatment. It should be noted that up to one-fourth of the patients showed response at the end of therapy though their serum creatinine level was not reduced by day 3. This may be due to increasing the dose of terlipressin in patients whom their serum creatinine level failed to reach an early reduction or showed a delayed renal response with respect to the improvement of hemodynamic status. In these patients, treatment with terlipressin was maintained after 3 days to achieve this delayed response effect. This finding is approved by Nazar et al. (2010).

The article "Endothelin-1/Nitric Oxide Ratio as a Predictive Factor of Response to Therapy With Terlipressin and Albumin in Patients With Type-1 Hepatorenal Syndrome" was published in 2020. Journal: Front Pharmacol.

In the current study, the 90-day survival probability in non-responders was 9% and in responders 40%. These results, in conjunction with the observation that patients with HRS where the albumin and terlipressin enhanced their renal capacity had marvelous posttransplantation results compared to patients without HRS (Restuccia et al., 2004), confirm that albumin plus terlipressin is a successful and helpful choice for HRS patients anticipating liver transplantation. The observations of this study were in accordance with previous reports which stated that type-1 HRS patients responding to therapy with albumin and terlipressin have longer survival expectancy compared to that of non-responders [(Ortega et al., 2002; Martín-Llahí et al., 2008; Neri et al., 2008; Sharma et al., 2008).

Moreover, to our knowledge, no studies published the role of changes in the ET-1/NO ratio as an independent predictor of response to albumin with terlipressin in type-1 HRS. Such results will certainly be much scrutinized, but there are some clear conclusions for the role of ET-1 and NO in the pathophysiology of HRS. Such findings add to our understanding and knowledge of the pathogenesis of HRS in a number of ways and provide a foundation for its management. This study's findings have a number of significant implications for future practice.

Of course, this study has some limitations that should be addressed. First, the sample size is small. Second, the current study is a single center study, and recruiting a large number of patients for such a meticulous study, is mandatory yet difficult due to the unavailability of terlipressin in many centers and type-1 HRS is not a common disorder. Third, the ET-1/NO ratio is not routinely measured in clinical practice. Furthermore, studies from multiple centers are needed to confirm these findings in HRS patients.

In conclusion, the outcomes of the current study, in type-1 HRS patients, indicate that a reduction in the ET-1/NO ratio and lower serum bilirubin baseline are considered good predictors of response to treatment with albumin and terlipressin. Future studies on treatment of type-1 HRS should discuss the possible mechanisms of declined response to pharmacological treatment and should search for new therapeutic options for non-responders.

The article "Endothelin-1/Nitric Oxide Ratio as a Predictive Factor of Response to Therapy With Terlipressin and Albumin in Patients With Type-1 Hepatorenal Syndrome" was published in 2020. Journal: Front Pharmacol.

## Data Availability Statement

The raw data supporting the conclusions of this article will be made available by the authors, without undue reservation, to any qualified researcher.

## Ethics Statement

The study was reviewed and approved by the Ethics Committee of Mansoura University, Egypt. (Proposal code: R.19.06.534). The patients/participants provided their written informed consent to participate in this study.

## Author Contributions

All the authors have accepted responsibility for the entire content of this submitted manuscript and approved submission. AA-R and NM acquired, analyzed and interpreted data; performed statistical analysis; and wrote, edited and reviewed the manuscript. MA, AA, and MT recruited and followed up with patients; acquired, analyzed and interpreted data; performed statistical analysis; critically revised the manuscript. AT recruited and followed up with patients; acquired, analyzed and interpreted data; critically revised the manuscript. AH recruited and followed up with patients; acquired, analyzed and interpreted data; critically revised the manuscript. RE acquired, analyzed and interpreted data; underwent laboratory investigations and revised the manuscript. WE and NE-W acquired, analyzed and interpreted data; performed statistical analysis; underwent laboratory investigations; critically revised the manuscript. All authors approved the final version of the article, including the authorship list.

## Conflict of Interest

The authors declare that the research was conducted in the absence of any commercial or financial relationships that could be construed as a potential conflict of interest.

## Abbreviations

HRS, hepatorenal syndrome; ET-1/NO ratio, endothelin-1/nitric oxide ratio; GFR, glomerular filtration rate; PMN, polymorphonuclear; SBP, spontaneous bacterial peritonitis; IVCCI, inferior vena cava collapsibility index; CBC, complete blood count; MELD, Model for End-Stage Liver Disease.
